The article "Eye Sign is an Alternative for Evaluation of the Microcirculation in Patients with Systemic Sclerosis" was retracted in 2023. Reasons: signs of a paper mill; suspected computer-generated content; unreliable results or conclusions; lack of ethics approval or compliance.

# Eye Sign is an Alternative for Evaluation of the Microcirculation in Patients with Systemic Sclerosis

**DOI:** 10.1155/2022/1034535

**Published:** 2022-11-04

**Authors:** Shujiao Yu, Xudong Ni, Jun Zhao, Rui Wu

**Affiliations:** ^1^Department of Immunlogy and Rheumatology, The First Affiliated Hospital of Nanchang University, Nanchang, China; ^2^Department of Biochemistry and Molecular Biology, Basic Medical Sciences, Nanchang University, Nanchang, China

## Abstract

**Objectives:**

To investigate consistency between eye sign and nailfold video capillaroscopy (NVC) in systemic sclerosis (SSc) patients and to evaluate eye sign with various parameters of disease and potential pulmonary involvement.

**Methods:**

A total of 60 SSc patients and 20 healthy individuals were enrolled. 20 SSc patients were complicated with pulmonary arterial hypertension (PAH); 20 SSc patients with interstitial lung diseases (ILD); 20 SSc patients without pulmonary involvement. All subjects were assessed using the methods of NVC and eye sign. Skin involvement was evaluated by modified Rodnan skin score (mRSS) and disease activity according to Medsger's severity score (MSS). Clinical manifestations and the presence of autoantibodies were carefully recorded. Any correlations between were evaluated with the Spearman correlation coefficient test.

**Results:**

According to the morphological changes revealed by NVC, 3 types of NVC patterns have been characterized (early pattern, active pattern, and late pattern). Eye sign showed distinguishing morphologic changes in three patterns of NVC and pulmonary involvements (PAH *vs* ILD) in SSc. A positive linear correlation was found between scores of eye sign and NVC in all patients with SSc (*r* = 0.629, *P*=0.001). A positive correlation of eye sign was found in all SSc patients with mRSS (*r* = 0.748, *P*=0.045) and MSS (*r* = 0.636, *P*=0.001).

**Conclusions:**

The study demonstrates that eye sign had a high consistency with NVC for the evaluation of the microcirculation in SSc patients and exhibited specific patterns in the early, active, and late phases of SSc. Eye sign can be used as a reliable method to classify and monitor SSc patients and replace the measurement of NVC.

## 1. Introduction

Systemic sclerosis (SSc) is a chronic multisystemic autoimmune disease characterized predominantly by fibrosis and widespread vascular disorders [1]. Microvascular damage occurs during the early stages of SSc and the ongoing vascular damage causes remodeling and disturbance of the capillary architecture, leading to microcirculation alterations [1–4]. In addition to the microvascular damage [5], SSc is associated with the damage of interstitial lung [6] and bone quality [7]. Nailfold videocapillaroscopy (NVC) is an effective tool of microcirculation examination, which is included in the 2013 guidelines of American College of Rheumatology (ACR) and European League Against Rheumatism (EULAR) for the preliminary classification of SSc [2]. So far, NVC has shown its undoubted value for the assessment and treatment of SSc [3]. According to the morphological changes revealed by NVC, 3 types of NVC patterns have been characterized: (1) an early pattern referred to as normal capillaries, with a well preserved capillary network containing only a few giant capillaries; (2) an active pattern revealed as the presence of numerous giant capillaries and hemorrhages, with only a minor decrease in capillary numbers; (3) a late pattern defined by severe loss of capillaries and extensive avascular areas; the capillary region appears disorganized and ramified and/or bushy capillaries are present [6, 7]. Three patterns of NVC reflect the different phases of SSc disease. Studies have shown an association between NVC and the extreme symptoms of SSc including PAH and ILD [8]. NVC is currently considered to be an excellent method to detect progression of SSc disease [6].

There are several regions of the human body where the systemic microcirculation can be directly observed, including the nail fold, bulbar conjunctiva, tongue, and lip. Compared to other regions, the bulbar conjunctiva is more stable and is influenced to a lesser extent by variations in temperature. However, complicated implementation has limited its application in clinical practice. Thus, eye sign, a simplified assessment of the bulbar conjunctiva microcirculation, was introduced into clinical practice in 1988 [9]. It characterizes 8 features of the microcirculation including enlarged and/or twisted capillaries, helical capillaries, ramified loops, microangioma, and hemorrhage (Figure 1 and Table 1). Previous studies have demonstrated that eye sign is a reliable and feasible assessment for blood stasis, disease activity, and organ involvement in rheumatic diseases [10]. Present research focused on NVC and ignored the role of bulbar conjunctiva microcirculation in SSc, while we discuss the consistency between eye sign and NVC in the evaluation of phase classifications, ongoing disease activity, and pulmonary involvement (PAH, ILD) in SSc patients in this study.

## 2. Patients and Methods

### 2.1. Enrolled Patients

The approval for the study was provided by the Medical Ethics Committee of the First Affiliated Hospital of Nanchang University (Ref.no: 2017016), and all patients received oral and written information and signed the informed consent form. Sixty SSc patients and 20 healthy subjects matched for gender and age were enrolled after providing written informed consent (Table 2). All patients met the 2013 ACR and EULAR criteria for the diagnosis of SSc [2]. Twenty patients with SSc had mild to moderate PAH with the average pulmonary artery pressure of 35–75 mm·Hg and without ILD. 20 SSc patients had mild and moderate ILD diagnosed by chest computerized tomography and impaired pulmonary function test with forced vital capacity (FVC) greater than or equal to 45% of normal and diffusing capacity of carbon monoxide (DLCO) greater than or equal to 30% of normal. As control group, 20 SSc patients without pulmonary involvement were included. Patients with fever, diabetes mellitus, hypertension, and eye conditions were excluded.

### 2.2. Methods

#### 2.2.1. Assessment of Eye Sign and Nailfold Capillaries

Each patient stayed for 30 min in a room maintained at a temperature of 18–25°C before examination. Eight eye signs were measured (both eyes) and scored by naked eye criteria (Table 1). Another operator performed NVC using a microcirculation detector with *a* × 200 contact lens. Nailfold capillaries of the distal row of fingers in both hands (excluding the thumbs) were examined. NVC microangiopathy patterns were assessed according to the classification previously described (*vide supra*). Giant and enlarged capillaries, capillary loss, microvascular disorganization, ramification of capillaries, and hemorrhage were the parameters evaluated to identify scleroderma patterns. A semiquantitative rating scale (range: 0–3) was used to score these altered microvascular parameters [11].

### 2.3. Autoantibody Test

Peripheral venous blood was taken and the titre of antinuclear antibodies (ANA) and anticentromere antibodies determined by indirect immunofluorescence. Anti-Scl 70 antibodies were characterized using ELISA.

### 2.4. Assessment of Skin Involvement and Disease Activity

mRSS was used and the sum of the scores used to assess involvement of the skin [12]. Clinical manifestations recorded included the presence of either limited (lcSSc) or diffuse (dcSSc) skin involvement was recorded. Disease severity was evaluated using the MSS [13].

### 2.5. Statistical Analysis

All statistical analyses were conducted with SPSS (ver. 22.0). Descriptive variables are given as the mean ± standard deviation (SD) and categorical data as percentages and numbers. Student's *t*-test was conducted to assess differences between 2 independent groups. ANOVA (*f*) and nonparametric tests were used for quantitative variables in more than 2 independent groups. Any correlations between were evaluated with the Spearman correlation coefficient test. *P* value < 0.05 were considered statistically significant.

## 3. Results

Systemic sclerosis patients were classified into early, active, or late groups according to the pattern of NVC. In the early group, the scores of eye sign appeared to be slightly increased but without a statistically significant difference compared to the control participants (*P* > 0.05). In contrast, scores in the active and late groups were much higher than in the early group and healthy subjects (*P* < 0.001) (Table 3). Although scores of eye sign was no significant difference between active and late group, specific morphologic changes were shown in two groups. In active group, eye sign predominantly showed enlarged capillaries, ramified loops, microangioma, and hemorrhage predominantly which align to changes of NVC in same patient (Figure 2). In late groups, twisted capillaries, microangioma, and wound spot were significantly frequent than other groups. No specific changes of eye sign found in early group.

A positive linear correlation was found between scores of eye sign and NVC in all patients with SSc (*r* = 0.629, *P*=0.001). A positive correlation of eye sign was found in all SSc patients with mRSS (*r* = 0.748, *P*=0.045) and MSS (*r* = 0.636, *P*=0.001).

Scores of eye sign in SSc patients with PAH or ILD were significantly greater than in patients without these conditions (Table 4). SSc patients with PAH showed frequent enlarged capillaries and hemorrhages while SSc-ILD patients presented with more twisted capillaries in the eye sign group compared to the PAH and control groups.

## 4. Discussion

Growing evidence suggests that peripheral microvascular changes reflect the degree of SSc, especially in those patients with life-threatening cardiopulmonary complications [9, 14]. A retrospective multicenter collaborative study of EULAR and EUSTAR databases revealed a significant correlation between vasculopathy and the involvement of various body organs [15]. Therefore, NVC is widely used in predicting SSc disease progression as the most common tool for evaluation of the systemic microcirculation. Our study found that eye sign had a linear correlation with the NVC score and also has its own specific 3 patterns in SSc, depending on the distinguished morphotic images of eye sign in the early, late, and active patterns of NVC. Furthermore, the scores of eye sign were positively correlated with mRSS and Medsger's disease severity score.

The findings in our study strongly suggest that eye sign can be used to monitor the progression of the disease and organ involvement. All the data suggests eye sign is a valuable tool as well as NVC in SSc diagnosis and treatment. Eye sign can directly observed by naked eye without need for instruments which make eye sign a convenient tool for clinicians.

It was reported in 1968 that bulbar conjunctival can become another place of microcirculation evaluation instead of nailfold microcirculation in rheumatic diseases [16]. A normal pattern in bulbar conjunctival microcirculation (BCM) consists of 3–5 vessels with dendritic shape in four areas around eyeball and venules range from 20 to 30 *μ*m while arterioles range from 10 to 20 *μ*m in diameter. The ratio of arteriole to venule is 1 : 2. Vascular structural damage and remodeling lead to enlarged capillaries, twisted capillaries, microhemorrhages, loss of capillaries, and angiogenesis [17, 18]. Eye sign was produced based on these typical changes in BCM. Our study showed the abnormalities of eye sign were presented in 92% (55/60) of SSc patients. Eye sign can be defined as early, active, late pattern, and NVC. Three pattern of eye sign might be defined that the “early” pattern refers to relatively normal capillaries morphology with a few twisted and enlarged vessels (<3); the “active” pattern is characterized with a few enlarged capillaries, increased ratio of deformity area of ramified loops to whole conjunctiva area and hemorrhage; the “late” pattern is characterized by severe twisted capillary with helical shape, microangioma, and numerous wound spot.

In conclusion, eye sign is feasible and convenient method in assessment of microvascular damage and disease activity in SSc patients. A few studies investigated the role of eye sign in SSc patients. The findings of our study supported that, in clinical practice, we may evaluate the activity and severity of SSc through eye sign in the future.

## Figures and Tables

**Figure 1:** Eye sign.

**Figure 2:** In active according to the pattern of NVC shows giant capillaries (blue arrow), hemorrhage (black arrows) in picture (a) while eye sign shows enlarged capillaries (blue arrow) and hemorrhage (black arrow) in picture (b). In late according to the pattern of NVC shows severe capillary loss with extensive avascular areas (orange arrow), disorganization of capillary area, and ramified capillaries (green arrow) in picture (c) while eye sign shows twisted capillaries (yellow arrows) and wound spot (red arrow) in picture (d).

**Table 1:** Scores of eye signs.

Characteristics	Score	
Enlarged capillaries	3–6	5
	>6	10

Twisted capillaries	3–6	5
	>6	10
Helical capillaries		10

Ratio of deformity area of ramified loops to the whole conjunctival area	1/8–1/4	5
	>1/4	10

Hemorrhages	1–3	5
	>3	10
Microangioma		10

Color tune of vessel and skin around eyelid	Mild	5
	Serious	10

Wound spot	1–2	5
	>3	10

**Table 2:** Baseline characteristics of SSc patients.

Variables	SSc (*n* = 60)	Early SSc	Late SSc	Active SSc
Age (years)	53.26 ± 11.60	49.56 ± 9.87	54.43 ± 10.56	51.18 ± 11.98
Sex (female)	35 (58.33)	6 (50)	19 (63.33)	10 (55.55)
Disease duration, months	30.73 ± 19.30	2.17 ± 1.25	46.07 ± 9.60	24.22 ± 9.99
BMI, kg/m^2^	24.21 ± 4.15	23.76 ± 3.98	24.86 ± 4.93	24.17 ± 4.22
Ranaud's phenomenon (%)	51 (85)	8 (66.67)	28 (93.33)	15 (83.33)
Scl type, *n* (%)				
Diffuse	26 (43.33)	3 (25)	16 (53.33)	7 (38.89)
Limited	34 (56.67)	9 (75)	14 (46.67)	11 (61.11)
Autoantibodies, *n* (%)				
ANA	28 (46.7)	4 (33.33)	17 (56.67)	7 (38.89)
Anti-scl-70	21 (35)	3 (25)	12 (40)	6 (33.33)
Anticentromere	16 (26.7)	3 (25)	9 (30)	4 (22.22)
ACA	9 (15)	1 (0.08)	6 (20)	2 (11.11)
mRSS, mean (SD)	15.95 ± 7.24	4.58 ± 1.51	21.23 ± 3.54	14.72 ± 4.16
MSS, mean (SD)	11.97 ± 4.60	4.25 ± 1.14	14.67 ± 2.51	12.61 ± 2.52
Score of eye sign	25.91 ± 7.51	17.08 ± 3.34	26.67 ± 4.98	29.72 ± 6.29
Score of NVC	7.82 ± 1.82	5.51 ± 1.86	8.46 ± 1.28	8.29 ± 1.32

**Table 3:** Eye sign in three phases of NVC.

	Early (*n* = 12)	Late (*n* = 30)	Active (*n* = 18)	Healthy (*n* = 20)	Early *vs* late	Early *vs* active	Late *vs* active
Total score	17.08 ± 3.34	27.83 ± 5.82	30.56 ± 4.16	14.75 ± 3.02	*P* < 0.001	*P* < 0.001	N/A
Enlarged capillaries	4.17 ± 1.95	4.67 ± 1.27	7.78 ± 2.56	3.50 ± 2.35	N/A	*P* < 0.001	*P* < 0.001
Twisted capillaries	3.75 ± 2.26	8.00 ± 2.49	3.89 ± 2.74	4.00 ± 2.05	*P* < 0.001	N/A	*P* < 0.001
Helical capillaries	0.00 ± 0.00	2.67 ± 4.49	1.67 ± 3.83	0.00 ± 0.00	*P*=0.003	N/A	N/A
Ramified loops	1.25 ± 2.26	0.67 ± 2.17	4.17 ± 3.92	1.00 ± 2.05	N/A	*P*=0.028	*P* < 0.001
Hemorrhages	1.67 ± 2.46	1.83 ± 2.45	5.83 ± 3.93	0.75 ± 1.83	N/A	*P*=0.003	*P* < 0.001
Microangioma	0.833 ± 1.95	3.00 ± 2.49	3.06 ± 3.04	0.50 ± 1.53	*P*=0.010	*P*=0.003	N/A
Color tune	2.08 ± 2.57	1.83 ± 2.78	2.50 ± 3.53	2.00 ± 2.51	N/A	*P*=0.033	N/A
Wound spots	2.50 ± 2.61	4.83 ± 2.78	2.22 ± 3.08	2.25 ± 2.55	*P*=0.017	N/A	*P*=0.004

Total score of early *vs* healthy, *P* > 0.05; total score of late *vs* healthy, *P* < 0.001; total score of active *vs* healthy, *P* < 0.001 .

**Table 4:** Eye sign in patients with PAH or ILD involvement.

	PAH (*n* = 20)	ILD (*n* = 20)	Control group^*∗*^ (*n* = 20)	PAH *vs* ILD	PAH *vs* control	ILD *vs* control
Total score	29.50 ± 5.60	29.25 ± 5.68	20.25 ± 5.25	N/A	*P* < 0.001	*P* < 0.001
Enlarged capillaries	7.00 ± 2.51	4.50 ± 2.34	4.75 ± 1.97	*P*=0.003	*P*=0.003	N/A
Twisted capillaries	3.75 ± 2.22	8.75 ± 2.22	5.25 ± 3.02	*P* < 0.001	N/A	*P* < 0.001
Helical capillaries	1.50 ± 3.66	4.00 ± 5.03	0.50 ± 2.24	N/A	N/A	*P*=0.007
Ramified loops	2.50 ± 3.44	1.50 ± 3.28	0.75 ± 1.83	N/A	N/A	N/A
Hemorrhages	5.75 ± 3.73	1.75 ± 2.44	1.25 ± 2.22	*P* < 0.001	*P* < 0.001	N/A
Microangioma	3.25 ± 2.94	2.00 ± 2.51	2.50 ± 2.56	N/A	N/A	N/A
Color tune	2.25 ± 3.43	2.50 ± 3.03	1.50 ± 2.35	N/A	N/A	N/A
Wound spots	3.25 ± 3.35	4.25 ± 3.35	3.25 ± 2.45	N/A	N/A	N/A

^*∗*^Control group:SSc patients without PAH and ILD.

## Data Availability

The data used to support the findings of this study are available from the corresponding author upon request.
